# Pathological changes in the maxillary sinus mucosae of patients with recurrent odontogenic maxillary sinusitis

This article has been retracted.

**DOI:** 10.12669/pjms.305.5312

**Published:** 2014

**Authors:** Lin Feng, Hua Li, Ling-Ling E, Chuan-Jie Li, Yan Ding

**Affiliations:** 1 Lin Feng, Department of Stomatology, Chinese PLA General Hospital, Beijing 100853, P. R. China.; 2 Hua Li, Department of Stomatology, Chinese PLA General Hospital, Beijing 100853, P. R. China.; 3 Ling-Ling E, Department of Stomatology, Chinese PLA General Hospital, Beijing 100853, P. R. China.; 4 Chuan-Jie Li, Department of Stomatology, Chinese PLA General Hospital, Beijing 100853, P. R. China.; 5 Yan Ding, Mitchell Medical Institute, University of South Alabama, Mobile, AL 36604, USA.

**Keywords:** Maxillary sinusitis, Mucosa, Odontogenic

## Abstract

***Objective: ***To study the structural and functional changes of maxillary sinus mucosae of patients with odontogenic maxillary sinusitis, and to improve the therapeutic effects.

***Methods:*** Ten mucosal biopsy samples collected during the surgeries of patients with recurrent odontogenic maxillary sinusitis were selected as Group A. Another ten mucosal biopsy sample were collected during retention cyst-removing surgeries and referred to as Group B. The mucosae were put in 10% neutral formalin solution for 1 day and prepared into 5-7 µm thick paraffin sections which were subjected to hematoxylin-eosin staining. The reactions included: (1) Reaction with T-lymphocyte (CD-3); (2) reaction with T-helper cell (CD-4); (3) reaction with T-suppressing cell (CD-8); (4) reaction with B-lymphocyte (CD-20). Polymeric horseradish peroxidase visualized detection system was used. The contents of CD3, CD4, CD8 and CD20 in the stained cells of the maxillary sinus mucosal layer were calculated. The responses of receptors to muramidase were classified as mild, moderate and strong. All data were analyzed by Statistica 6.0 package for Windows based on Mann-Whitney non-parametric standards.

***Results:*** The epithelial tissues in the maxillary sinus mucosa of Group B were covered with multiple rows of cilia. The epithelial cells of Group A suffered from degeneration, shrinkage and desquamation. Different cells were distributed in the autologous mucosal layer, of which macrophages, fibroblasts, lymphocytes and neutrophils were dominant. The average contents of macrophages and lymphocytes accounted for 42.8%. Lymphocyte subset analysis showed that the number of CD3 cells exceeded that of CD20 ones and there were more CD4+ cells than CD8+ ones. T-helper and T-suppressing cells were distributed remarkably differently. CD8+ cells were mainly located inside and under the epithelium, while CD4+ cells were scattered in the autologous matrix.

***Conclusion:*** For patients with recurrent odontogenic maxillary sinusitis, the maxillary sinus mucosa mainly suffered from regeneration of epithelial tissues and inhibition of cell proliferation, which were accompanied by damages to the protective and shielding effects of the mucociliary transport system. Macrophages and lymphocytes dominated in the infiltration of autologous mucosal layer, and the coexisting copious fibroblasts indicated the onset of inflammation.

## INTRODUCTION

Odontogenic maxillary sinusitis accounts for 10-12% of the total cases.^1^ Maxillary sinus is prone to odontogenic infections due to expansion of long-term, chronic apical periodontitis, radicular cyst, odontogenic jaw cyst, intrusion of apparatus or root canal filling materials, invasion of surgical dental extraction-induced residual tooth root, dental implant-induced maxillary sinus augmentation, and even "Le-fort" maxillary osteotomy.^1^^,^^2^

The postoperative recurrence rate of odontogenic maxillary sinusitis is as high as 80%^3^ because it is commonly treated by aggressive protocols without considering bone tunnel complex, nasal septum or mucociliary transport system**.**^4^ However, mucociliary functions are determined by ciliated epithelium and the matrix of maxillary sinus mucosa.^5^ Despite some clinical studies, the pathological characteristics of recurrent odontogenic maxillary sinusitis should be clarified. Therefore, we studied the structural and functional changes of the maxillary sinus mucosae of patients with recurrent odontogenic maxillary sinusitis, aiming to improve the therapeutic outcomes.

## METHODS

This study has been approved by the institutional ethics committee of our hospital, and written consent has been obtained from all enrolled subjects. Ten mucosal biopsy samples collected during the surgeries of patients with recurrent odontogenic maxillary sinusitis in 2013 were used as the study materials and referred to as Group A (Fig.1). The patients had received maxillary sinus surgeries 6-18 months before this study. Another ten mucosal biopsy sample were collected during retention cyst-removing surgeries in 2013 and referred to as Group B. The patients were 17-26 years old (mean: 23.83 ± 2.51). The mucosae were put in 10% neutral formalin solution for 1 day and prepared into 5-7 µm thick paraffin sections which were subjected to hematoxylin-eosin staining. Histochemical study was performed according to standard methods. The reactions included: (1) Reaction with T-lymphocyte (CD-3); (2) reaction with T-helper cell (CD-4); (3) reaction with T-suppressing cell (CD-8); (4) reaction with B-lymphocyte (CD-20).

Antibodies for CD3, CD8, CD20 and muramidase (Mur) were purchased from Dako (Denmark), and that for CD4 was obtained from Novocastra (UK). Polymeric horseradish peroxidase visualized detection system was used (BioGenex). The contents of CD3, CD4, CD8 and CD20 in the stained cells of the maxillary sinus mucosal layer were calculated (%). The responses of receptors to Mur were classified as mild, moderate and strong.^5^ All data were analyzed by Statistica 6.0 package for Windows based on Mann-Whitney non-parametric standards.

## RESULTS

The contents of stained CD3, CD4, CD8 and CD20 cells and the Mur activity in maxillary sinus mucosa are listed in Table-I. The lymphocyte subset analysis showed that the number of CD3 cells was higher than that of CD20 ones and there were more CD4+ cells than CD8+ ones.

Blood vessels around the autologous mucosal layer were infiltrated with aggregated CD3+ cells (Fig.2-1). T-helper and T-suppressing cells were distributed distinctively differently. CD8+ cells were mainly distributed inside and under the epithelium (Fig.2-2), and CD4+ cells were scattered in the autologous matrix (Fig.2-3).

## DISCUSSION

It is not very difficult to diagnose odontogenic maxillary sinusitis in clinical practice.^6^ Generally, CT examination of maxillary tooth discloses increase of sinus density or thickening of mucosa. Meanwhile, CT examination, which discloses microstructures of soft and bone tissues, can clarify the relationship between cysts and maxillary sinus wall defects and position foreign materials accurately, thus becoming a crucial evidence for diagnosing odontogenic maxillary sinusitis.^7^^,^^8^ Moreover, CT examinations at axial, sagittal and coronal planes clearly show the intrusion ranges of periapical cysts into maxillary sinus and the injuries of anterolateral wall, which provide valuable evidence for surgeries by helping determine the pathological changes beforehand. Odontogenic maxillary sinusitis is pathologically manifested as chronic inflammation complicated with polyps and lining of cyst wall with stratified squamous epithelium.^9^^,^^10^

**Fig.1:** Endoscopic image of maxillary sinus mucosa sample from

Group A (1), X-ray images at Water’s position (2 and 3), and MRI image (4).

**Fig.2:** Destruction of cells in maxillary sinus mucosa. 1: Sample A-2, infiltration of autologous mucosal layer by CD3+ cells (with CD3- antibody, stained by benzidine and hematoxylin); 2: sample A-5, distribution of CD8+ cells inside and under the epithelium (with CD8- antibody, stained by benzidine and hematoxylin); 3: sample A-9, CD4+ cells in autologous mucosal layer (with CD4- antibody, stained by benzidine and hematoxylin).

**Table-I:** Contents of stained CD3, CD4, CD8 and CD20 cells and Mur activity in maxillary sinus mucosa

***Item***	***Group A (N=10)***	***Group B (N=10)***
CD3 (%)	16.42±2.90	6.81±2.08*
CD4 (%)	9.88±1.15	4.97±1.40*
CD8 (%)	4.64±1.11	1.84±0.68*
CD20 (%)	2.25±0.44	2.3±0.58
Mur	69.33±9.81	57.31±17.10

* P<0.05.

Under pathological conditions, the maxillary sinus mucosa is evidently thickened compared with normal one, which is associated with chronic inflammation-induced mucosal layer edema (mostly for the youth), cell infiltration and connective tissue hyperplasia (mostly for the elderly).^11^ The depth of maxillary sinus mucosal epithelium gradually decreases with aging, which can be attributed to the attenuated cell regenerability after long-term external stimulation.^12^ In addition, mucosal edema is affected by gender and age^13^ owing to the infiltration of exudates from different connective tissues. The degree of edema is not related with position. Probably, long-term inflammation involves the mucosae of different sinus walls, which increases the capillary permeability, thus enabling granulation and then fibrosis.^14^^,^^15^

In this study, the epithelial tissues in the maxillary sinus mucosae of Group B were covered with multiple rows of cilia. In contrast, the epithelial cells of Group A were subjected to degeneration, shrinkage and desquamation. In a part of epithelial layers, glass-like cells proliferated, and there was transition from multiple rows of epithelial tissues to single-layer three-dimensional ones because of cilium missing. Various cells were distributed in the autologous mucosal layer, of which macrophages, fibroblasts, lymphocytes and neutrophils were dominant. Particularly, the average contents of macrophages and lymphocytes accounted for 42.8%. Lymphocytes were concentrated in the autologous matrix, with a small amount of them infiltrating and aggregating in the regions under the epithelium. The lymphocyte subset analysis showed that the number of CD3 cells was higher than that of CD20 ones and there were more CD4+ cells than CD8+ ones. In this case, CD3+ cells aggregated and infiltrated around the blood vessels in the autologous mucosal layer. T-helper and T-suppressing cells were distributed apparently differently. CD8+ cells were mainly located inside and under the epithelium, whereas CD4+ cells were scattered in the autologous matrix. CD8+ cells appeared inside the epithelium of patients with recurrent maxillary sinusitis due to the cytotoxicity of destructed cells, accompanied by degeneration of epithelial layer, tissue deformation and damages of mucociliary transport functions. Although the content of CD4+ cells in the mucosa significantly exceeded that of Group B, the ratio of CD4 cells to CD8 ones at 2.1:1 (standard: 2.7:1) verified that the preventive effects of mucosa were weakened, which was also demonstrated by the low activity of Mur in macrophages. In the meantime, such destructions may lead to long-term inflammation and even hardening of autologous mucosal layer. The results were associated with the activity of macrophages and the increase of fibroblast growth factor.

Hence, the maxillary sinus mucosa mainly suffered from regeneration of epithelial tissues and suppression of cell proliferation, which were concomitant with damages to the protective and shielding effects of the mucociliary transport system. Macrophages and lymphocytes predominated in the infiltration of autologous mucosal layer, and the resultant copious fibroblasts simultaneously suggested the onset of inflammation.

## Authors Contributions:

**HL and LF:** Designed the protocol and prepared the final manuscript.

**LLE, CJL** **and** **YD** **: **Clinical data collection and experiments.
